This article has been retracted.

# The Efficacy of Calcium Carbonate-Vitamin D3 in Pregnant Women for the Prevention of Hypertensive Disorders in Pregnancy

**DOI:** 10.1155/2022/7971976

**Published:** 2022-08-11

**Authors:** Zhen Chen, Jing Chen

**Affiliations:** Department of Maternal and Child Health Care, Shiyan Maternal and Child Health Hospital, Shiyan, Hubei, China

## Abstract

**Objective:**

To evaluate the efficacy of calcium carbonate-vitamin D3 in pregnant women for the prevention of hypertensive disorders in pregnancy.

**Methods:**

Between April 2020 and June 2021, 60 pregnant women undergoing prenatal examinations in our hospital were recruited and assigned via the random number table method at a ratio of 1 : 1 to receive conventional pregnancy care (observation group) or conventional pregnancy care plus calcium carbonate-vitamin D3 administration (experimental group). Outcome measures included blood pressure, blood calcium, the occurrence of hypertensive disorders, and adverse events.

**Results:**

The diastolic blood pressure (DBP) and systolic blood pressure (SBP) levels at delivery in the experimental group were significantly lower than those in the observation group (*P* < 0.05). Pregnant women in the experimental group had significantly higher blood calcium levels at labor than those in the observation group (*P* < 0.05). The administration of calcium carbonate-vitamin D3 resulted in a significantly lower incidence of hypertensive disorders and adverse events versus conventional pregnancy care (*P* < 0.05).

**Conclusion:**

The effect of calcium carbonate-vitamin D3 administration during pregnancy for the prevention of hypertensive disorders is significant, which effectively improves the blood calcium level of pregnant women and reduces the occurrence of adverse events, so it is worthy of clinical promotion and application.

## 1. Introduction

Hypertensive disorder of pregnancy is a syndrome unique to pregnancy, which mainly occurs after 20 weeks of gestation. The disease mainly presents clinical symptoms such as edema and hypertension, and it is easy to complicate with multiple organ dysfunction, resulting in poor maternal and infant outcomes. Studies have pointed out that the incidence of gestational hypertension in China is as high as 9.7% to 10.4%, which poses immense threat to maternal and infant health [1, 2]. The gestational hypertension can be classified into the categories of “sub-halo,” “sub-swollen,” and “eclampsia” with the liver-kidney yin deficiency and liver-yang hyperactivity. The liver-kidney yin deficiency type is one of the most common clinical syndromes. Most of the patients are vulnerable to deficiency of liver and kidney yin in the body due to lack of congenital development. It is known that kidney stores essence, liver stores blood, with essence and blood sharing with the same origin. During pregnancy, if the essence and blood are injected to nourish the fetus, in the second and third trimesters of pregnancy, the kidney yin deficiency is often manifested, and the yin deficiency is insufficient to restrain the yang, inducing gestational hypertension. Therefore, the main principles of treatment are to nourish the yin of the liver and kidney, and to suppress the yang of the liver [3, 4].

Hypertensive disorder of pregnancy, together with bleeding and infection, constitutes the three fatal pregnancy complications, and becomes one of the main causes of maternal death. At present, the specific pathogenesis of gestational hypertension is elusive, but calcium deficiency is mostly believed to be a major contributor to gestational hypertension [5]. Epidemiological studies have found that the incidence of gestational hypertension in calcium-deficient people is significantly higher than that in healthy people [6]. Pregnant women's blood volume expansion, increased calcium excretion, and the inhibitory effect of progesterone on calcium absorption result in a decrease in serum calcium levels. In recent years, with the improvement of people' understanding of the function of calcium in human physiology, it is believed that the occurrence of gestational hypertension may be associated with calcium [7]. Clinical research has found that the calcium requirement of the maternal body increases significantly at about 20 weeks of gestation [8], and at about 30 weeks, the calcium requirement of the maternal body can be about 6 times higher than that at 20 weeks, so the maternal body is prone to calcium deficiency in the second trimester [9].

Calcium deficiency in the maternal organism increases the permeability of cell membranes and causes a significant increase in the concentration of calcium ions in the vascular smooth muscle cells, which predisposes to hypertensive disorders during pregnancy [10]. The maternal body is the only source of calcium and nutrition for the fetus, and deficiency of calcium in the maternal body leads to calcium deficiency in the fetus, which seriously compromises the maternal health and the normal growth and development of the fetus [11]. Calcium carbonate-vitamin D3 tablets are a compound calcium supplement commonly used in clinical practice to rapidly replenish calcium in the body, and clinically relevant research has indicated no toxic side effects of the drug on pregnant women and fetuses [5].

In the present study, 60 pregnant women undergoing prenatal examinations in our hospital were recruited between April 2020 and June 2021 to evaluate the efficacy of calcium carbonate-vitamin D3 in pregnant women for the prevention of hypertensive disorders in pregnancy and provide a clinical reference.

## 2. Materials and Methods

### 2.1. Baseline Data

Between April 2020 and June 2021, 60 pregnant women undergoing prenatal examinations in our hospital were recruited and assigned via random number table method at a ratio of 1 : 1 to an observation group or an experimental group.

The participants provided the informed consent form before enrollment, and the study protocol was granted by the hospital ethics committee (SD-SDE20200402). All procedures were in compliance with the guidelines of the Declaration of Helsinki.

### 2.2. Inclusion and Exclusion Criteria

Inclusion criteria: (1) All subjects included in this study were diagnosed with gestational hypertension through relevant examinations. (2) Complete medical history data. (3) Did not receive any treatment for gestational hypertension previously. (4) The patient's mental cognition is normal and can cooperate with the medical staff to complete the whole treatment.

Exclusion criteria: (1) with hypertension, diabetes mellitus, and liver and kidney insufficiency before this diagnosis; (2) with severe mental illness; (3) with malignant tumor; (4) with infectious diseases; (5) with a history of antihypertensive treatment.

### 2.3. Methods

Pregnant women in the observation group received a reasonable diet and exercise interventions to help them control their body mass, without the administration of calcium supplements. Pregnant women in the experimental group received 1.5 g calcium carbonate-vitamin D3 (Beijing Kangyuan Pharmaceutical Co., Ltd., Approval No. H20090334) orally, twice daily, and the treatment was continued until the delivery [12].

On the basis of the treatment in two groups, patients were given Qiju Dihuang Decoction with modified and subtracted treatment. The ingredients of the prescription were 2 g of whole scorpion, 12 g of herb of *Herba cirsii*, *Cirsium japonicum* dc, and turtle shell, respectively, 15 g of *Ophiopogon japonicus*, mulberry seed, and Scrophularia Radix, respectively, 10 g of chrysanthemum, salvia, earthworm, red peony root, angelica, *Rehmannia glutinosa*, and wolfberry, and 30 g of mother of pearl, cassia, oyster, and keel, respectively. It was boiled in water to take 500 mL of juice, and taken with warm water in the morning and evening, for a total of 2 weeks.

### 2.4. Outcome Measures

1. Blood pressure level: the diastolic blood pressure (DBP) and systolic blood pressure (SBP) levels were measured upon enrollment and at labor using the EK648 electronic blood pressure monitor purchased from Shanghai Yuejin Medical Equipment Co.
2. Blood calcium level: 1 ml of elbow venous blood was collected from pregnant women upon enrollment and at the time of delivery and stored at 4°C for assay. Before and after the treatment, the fasting serum was secured and determined in the morning by the rate method (Beckman brand automatic biochemical analyzer produced by Beckman Coulke, USA).
3. Incidence of hypertensive disorders during pregnancy: the occurrence of hypertensive disorders was recorded by the medical staff of our hospital as per the following criteria: the pregnant woman had the first episode of elevated blood pressure during pregnancy with a systolic blood pressure ≥140 mmHg or diastolic blood pressure ≥90 mmHg.
4. Adverse events: adverse events including joint pain, low back pain, gastrocnemius spasm, and numbness of the limbs were recorded.

### 2.5. Statistical Analysis

The data obtained in this study were analyzed using the SPSS21.0 software, and GraphPad Prism 8 was used to plot the graphics. The measurement data are expressed as (mean ± SD) and analyzed using the Student's *t*-test after the test of normal distribution, and the count data are expressed as cases (%) and analyzed using the chi-square test. Differences were considered statistically significant at *P* < 0.05.

## 3. Results

### 3.1. Baseline Patient Profile

The baseline characteristics of the observation group (aged 22–34 years), body mass of 51–76 kg, gestational week of 20–27) weeks, were comparable with those of the experimental group (aged 21–35 years, body mass of 50–75 kg, gestational week of 21–27 weeks) (*P* > 0.05) (Table 1).

### 3.2. Blood Pressure

The DBP and SBP levels at delivery in the experimental group were significantly lower than those in the observation group (*P* < 0.05) (Figure 1).

### 3.3. Blood Calcium Levels

Pregnant women in the experimental group had significantly higher blood calcium levels at labor than those in the observation group (*P* < 0.05). (Figure 2).

### 3.4. Incidence of Hypertensive Disorders and Adverse Events

The administration of calcium carbonate-vitamin D3 resulted in a significantly lower incidence of hypertensive disorders and adverse events versus conventional pregnancy care (*P* < 0.05) (Table 2).

## 4. Discussion

The nutritional requirements and intake of pregnant women are significantly higher compared to nonpregnant women of the same age [13, 14]. Hypertensive disorders in pregnancy are specific to women during pregnancy and mostly occur after 20 weeks of gestation. The clinical manifestations of the disease include hypertension, edema, and proteinuria, and some severe cases may experience nausea, vomiting, abdominal pain, convulsions, and coma [15], which severely compromise the health of the mother and fetus. At present, Western medicine treatment mainly focuses on blood pressure, sedation, volume expansion, and spasmolysis. Clinically, patients often receive nifedipine sustained-release tablets, which is a calcium channel blocker, and can effectively reduce the entry of calcium ions into cells through the slow calcium channel, reduce the excitation of blood vessels, reduce the resistance of blood vessels, and then achieve the purpose of antihypertension. However, the long-term use of the drug is associated with many adverse reactions that easily increase the physical and mental burden of the patient [16].

Clinical research has shown that hypertensive disorders during pregnancy are mainly attributed to calcium deficiency [17]. The metabolic demand of pregnant women and the growth and development of the fetus increase significantly during pregnancy, during which the unfulfilled calcium demand of the pregnant women predisposes to the development of hypertensive disorders [18]. Research has shown that calcium deficiency in pregnant women causes abnormal contraction of vascular smooth muscle, leading to an increase in blood pressure and an increased risk of hypertensive disorders during pregnancy [19]. Calcium carbonate-vitamin D3 tablets are a compounded calcium supplement commonly used in clinical practice [20], consisting of calcium carbonate and vitamin D3. Vitamin D3 is a fat-soluble vitamin that efficiently promotes the absorption and utilization of calcium elements in pregnant women, reduces the metabolism of calcium elements by the kidneys, and helps maintain the blood calcium level in the body [21]. Wang[22] et al. stated that the detection of blood pressure levels in the maternal organism is effective in preventing the occurrence of hypertensive disorders [23].

The ingredients of the prescription were 2 g of whole scorpion, 12 g of herb of *Herba cirsii*, *Cirsium japonicum* dc, and turtle shell, respectively, 15 g of *Ophiopogon japonicus*, mulberry seed, and Scrophularia Radix, respectively, 10 g of chrysanthemum, salvia, earthworm, red peony root, angelica, *Rehmannia glutinosa*, and wolfberry, and 30 g of mother of pearl, cassia, oyster, and keel, respectively. It was boiled in water to take 500 mL of juice, and taken with warm water in the morning and evening, for a total of 2 weeks.

From the perspective of traditional Chinese medicine, gestational hypertension is mostly related to the deficiency of liver and kidney, deficiency of qi and blood, and imbalance of yin and yang in pregnant women. Its treatment should focus on nourishing yin and clearing heat, and calming liver and subduing yang. The patients were given Qiju Dihuang Decoction on the basis of conventional Western medicine treatment. Among the prescription ingredients, herb of *Herba cirsii* has the effect of strengthening the heart and inhibiting blood vessels. *Cirsium japonicum* dc and red peony can remove blood stasis and reduce swelling. Oyster can enhance the antihypertensive, clearing heat and sedative effects of the prescription. Mother-of-pearl and keel have the effect of calming the liver and subduing the yang. The combination of various medicines can effectively improve the symptoms of patients with hypertension, edema, proteinuria, etc., and can effectively protect the function of the body's organs and achieve the purpose of treatment.

In the present study, the result showed that the DBP and SBP levels at delivery in the experimental group were significantly lower than those in the observation group, indicating that the administration of calcium carbonate-vitamin D3 tablets during pregnancy can effectively contribute to the reduction and control of blood pressure levels in pregnant women. The reason may be that the administration of calcium carbonate-vitamin D3 alleviates the abnormal contraction of maternal vascular smooth muscle, thereby providing effective control of maternal blood pressure levels [24]. Calcium deficiency is the main cause of hypertensive disorders in pregnancy, and there are several reasons for calcium deficiency: (1) the blood volume of the pregnant woman's body will increase significantly during pregnancy, which may lead to a decrease in the blood calcium level [25]. (2) The glomerular filtration rate of pregnant women increases during pregnancy, resulting in a large amount of calcium excreted in the urine and a decrease in the blood calcium level of the maternal organism [26]. (3) The level of progesterone in the body of pregnant women increases during pregnancy, and the high level of progesterone inhibits the absorption of calcium elements in the body, which contributes to the reduction of blood calcium levels in the body of pregnant women [27]. Here, pregnant women in the experimental group had significantly higher blood calcium levels at labor than those in the observation group, suggesting that the administration of calcium carbonate-vitamin D3 during pregnancy can effectively increase blood calcium levels in the body. The reason may be that vitamin D3 effectively promotes the absorption and utilization of calcium elements in pregnant women, facilitating the improvement and maintenance of blood calcium levels [28, 29]. Moreover, the administration of calcium carbonate-vitamin D3 resulted in a significantly lower incidence of hypertensive disorders and adverse events versus conventional pregnancy care, indicating a safety benefit of calcium carbonate-vitamin D3 for the prevention of hypertensive disorders by lowering the risk of hypertension during pregnancy.

Preventive calcium supplementation during pregnancy has been a clinical consensus, but due to factors such as health literacy and economic conditions, pregnant women have poor compliance with treatment and often fail to achieve ideal preventive effects. Although this study provides a certain guiding significance for calcium supplementation treatment for patients with gestational hypertension, there are still the following problems: the number of samples is small, the observation period is short, and there is no long-term follow-up. It is hoped that in the future, the majority of researchers and patients will cooperate to conduct clinical studies with larger samples, so as to provide more clinical evidence for the research and application.

To summarize, the effect of calcium carbonate-vitamin D3 administration during pregnancy for the prevention of hypertensive disorders is significant, as it effectively improves pregnant women's blood calcium levels and reduces the occurrence of adverse events, making it worthy of clinical promotion and application.

## Figures and Tables

**Figure 1:** Comparison of blood pressure ($\bar{x}$ ± s).  ^*∗*^*P* < 0.05.

**Figure 2:** Comparison of blood calcium levels ($\bar{x}$ ± s).  ^*∗*^*P* < 0.05.

**Table 1:** Comparison of baseline data (*n* (%)).

	Observation group (*n* = 30)	Experimental group (*n* = 30)	*t* or *x*^2^	*P* value
Age (year)	$\bar{x}$ ± s	$\bar{x}$ ± s		
Mean age (year)	26.12 ± 3.15	26.28 ± 3.16	−0.196	0.845
Body mass (kg)	$\bar{x}$ ± s	$\bar{x}$ ± s		
Mean body mass (kg)	64.51 ± 6.78	64.39 ± 6.68	0.069	0.945
Gestational week (week)	$\bar{x}$ ± s	$\bar{x}$ ± s		
Mean gestational week (week)	24.32 ± 1.27	24.27 ± 1.33	0.149	0.882

**Table 2:** Comparison of incidence of hypertensive disorders and adverse events (*n* (%)).

	Observation group (*n* = 30)	Experimental group (*n* = 30)	*x* ^2^	*P* value
Incidence of hypertensive disorder	9 (30%)	1 (3%)	7.68	0.006
Adverse events				
Joint pain	3	1		
Low back pain	2	0		
Gastrocnemius muscle spasm	2	0		
Numbness of limbs	3	1		
Total incidence (%)	10 (33%)	2 (7%)	6.667	0.01

## Data Availability

No data were used to support this study.
